This article has been retracted.

# Activation of Akt1 accelerates carcinogen-induced tumorigenesis in mammary gland of virgin and post-lactating transgenic mice

**DOI:** 10.1186/1471-2407-14-266

**Published:** 2014-04-17

**Authors:** Yanyuan Wu, Juri Kim, Yayha Elshimali, Marianna Sarkissyan, Jaydutt V Vadgama

**Affiliations:** 1 Division of Cancer Research and Training, Charles R. Drew University of Medicine and Science, 1731 East 120th Street, Los Angeles, CA 90059, USA; 2 Jonsson Comprehensive Cancer Center and David Geffen UCLA School of Medicine, Los Angeles, CA, USA

**Keywords:** Myr-Akt1, Tumorigenesis, Mammary gland, Estrogen, Lactation, Breast cancer

## Abstract

**Background:**

Data from *in vivo* and *in vitro* studies suggest that activation of Akt regulates cell survival signaling and plays a key role in tumorigenesis. Hence, transgenic mice were created to explore the oncogenic role of Akt1 in the development of mammary tumors.

**Methods:**

The transgenic mice were generated by expressing myristoylated-Akt1 (myr-Akt1) under the control of the MMTV-LTR promoter. The carcinogen 7, 12 dimethyl-1,2-benzanthracene (DMBA) was used to induce tumor formation.

**Results:**

The MMTV driven myr-Akt1 transgene expression was detected primarily in the mammary glands, uterus, and ovaries. The expression level increased significantly in lactating mice, suggesting that the response was hormone dependent. The total Akt expression level in the mammary gland was also higher in the lactating mice. Interestingly, the expression of MMTVmyr-Akt1 in the ovaries of the transgenic mice caused significant increase in circulating estrogen levels, even at the post-lactation stage. Expression of myr-Akt1 in mammary glands alone did not increase the frequency of tumor formation. However, there was an increased susceptibility of forming mammary tumors induced by DMBA in the transgenic mice, especially in mice post-lactation. Within 34 weeks, DMBA induced mammary tumors in 42.9% of transgenic mice post-lactation, but not in wild-type mice post-lactation. The myr-Akt1 mammary tumors induced by DMBA had increased phosphorylated-Akt1 and showed strong expression of estrogen receptor (ERα) and epidermal growth factor receptor (EGFR). In addition, Cyclin D1 was more frequently up-regulated in mammary tumors from transgenic mice compared to tumors from wild-type mice. Overexpression of Cyclin D1, however, was not completely dependent on activated Akt1. Interestingly, mammary tumors that had metastasized to secondary sites had increased expression of Twist and Slug, but low expression of Cyclin D1.

**Conclusions:**

In summary, the MMTVmyr-Akt1 transgenic mouse model could be useful to study mechanisms of ER-positive breast tumor development.

## Background

The serine/threonine kinase Akt, also known as Protein Kinase B (PKB) plays a key role in multiple cellular processes. To date, three human isoforms of Akt have been identified: Akt1/PKBα, Akt2/PKBβ and Akt3/PKBγ [1]. Akt1 has been shown to play a key role in cellular survival pathways by inhibiting apoptotic processes, inducing cell proliferation, and protein synthesis [1-3]. The PKB/Akt pathway can be activated by a variety of growth factors, hormones, and cytokines [4,5] and can participate in oncogenic transformation of mammalian cells through its regulation of key biological process [6,7]. Akt is frequently constitutively active in many types of human cancers, such as breast, ovarian, and prostate [8-10]. It has been demonstrated by our group and others that activated Akt1 in tumor cells are associated with high grade tumors, late stage of diagnosis, and poor outcome in patients [9,10]. Cell lines derived from breast cancer patients who were resistant to trastuzumab treatment have also shown upregulation of Akt [11]. Furthermore, patients who have poor outcome and resistance to endocrine therapy have also been found to have activated Akt1 in their tumor cells [9]. We have recently demonstrated that activation of Akt1 in breast tumor cells *in vitro*, leads to inactivation of FOXO1 and a decrease in response or resistance to trastuzumab-induced growth inhibition in HER2 overexpressing breast cancer cells [12]. Significant data from *in vivo* and *in vitro* studies suggest that activation of Akt regulates cell survival signaling and plays a key role in tumorigenesis. Although a few *in vivo* studies have explored the role of Akt in normal mammary development and tumorigenesis using transgenic mouse models [13-16], the mechanisms associated with the oncogenic role of Akt remains to be further elucidated.

In this study, a transgenic mouse model with activated Akt was developed, such that the *in vivo* mechanisms by which Akt induces tumor development and progression in the mammary gland can be better understood. This transgene model also explores the mechanisms by which a carcinogen, DMBA, may further enhance the induction of Akt1 driven mammary gland tumors in virgin and post-lactation mice. In addition, this MMTVmyr-Akt1 transgenic model could serve as a preclinical model for studying ER-positive breast cancers that become resistant to endocrine therapy and develop into metastatic disease. Specifically, this model could be used to develop novel target therapies in breast cancer research and treatment.

## Methods

This study was approved by Institutional Animal Care and Use Committee (IACUC) at Charles R. Drew University of Medicine and Science.

### Generation of transgenic mice

The DNA structures of constitutively active Akt1 (myr-Akt1) (#21-151) were obtained from the Upstate Biotechnology Company. The activation of Akt1 was accomplished by the presence of the 11 N-terminal amino acids of avian c-*src* that were required for protein myristoylation at the amino terminus of Akt1. The promoter in the original myr-Akt1 DNA structure (#21-151, Upstate Biotechnology) was a human cytomegalovirus immediate-early promoter (CMV). To create a mammary tissue specific mouse transgene, the CMV promoter was replaced by the MMTV-LTR (American Type Culture Collection). The MMTV-LTR promoter was inserted into plasmid DNA containing myr-Akt1 sequences (Additional file 1: Figure S1A). The construct was digested and the fragments containing the MMTV-LTR promoter, myr-Akt1 sequences, and SV40 polyadenylation signal were isolated and purified (Additional file 1: Figure S1B). The transgenic mice were generated by microinjection of DNA directly into one of the pronuclei of C57BL/6 mouse-fertilized zygotes at the University of California, at Los Angeles (UCLA) transgenic facility. The genotyping of the transgenic MMTVmyr-Akt1 mice was performed by polymerase chain reaction (PCR) with genomic DNA extracted from the tails of mice. Integration of the transgene and the transgene copy number were determined by real-time quantitative PCR [17,18]. The standard curve was generated by mixing non-transgenic tail DNA with transgene plasmid DNA. The single copy transgene was determined using the calculation method provided by the University of Michigan Transgenic Animal Model Core facility available at http://www.med.umich.edu/tamc. An example of the copy number standard curve is shown in Additional file 1: Figure S1C. The Ct numbers from the genomic DNA of positive transgenic and wild-type (WT) litters were filled into a linear regression model and the copy number of transgenes was estimated. As shown in Additional file 1: Figure S1D, myr-Akt1+/+was defined as mice with 2 copy numbers of the transgene, such as mice 2-11 and 2-23. Myr-Akt1+/- was defined as mice with 1 copy number of the transgene, such as mice 2-10, 2-12, and 2-33. Mice 2-14 and 2-21 were transgene negative.

### DMBA Treatment

The carcinogen 7, 12 dimethyl-1,2-benzanthracene (DMBA, Sigma) was dissolved in olive oil at a concentration of 10 mg/ml. This mixture was heated at 37°C and shaken vigorously to fully dissolve the DMBA. Virgin and post-lactation female transgenic (MMTVmyr-Akt1+) and wild-type (WT) mice were treated with 1 mg doses of DMBA *via* oral gavage weekly for a total of 6 weeks. Mice were maintained in the absence of males and were checked by palpation for tumor formation after completion of the DMBA treatments. The mice were sacrificed by CO2 inhalation either when tumors reached 225 mm^2^ or if the mice became moribund either during or at the end of the 34 week observation period. As indicated before, this study was approved by Institutional Animal Care and Use Committee (IACUC) at Charles R. Drew University of Medicine and Science.

### Histopathology and immunohistochemistry (IHC)

The mammary glands, tumor tissues, and other organs from the mice were formalin-fixed and embedded in paraffin. The tissue sections were stained with either hematoxylin and eosin (H&E) or underwent immunohistochemistry (IHC) with specific antibodies. The antibodies used were as follows: anti-phospho-Akt1(ser473) (Cell Signaling, MA), anti-pan-keratins (pan-CKs), anti-ERα, anti-EGFR (Santa Cruz Biotechnology, CA), and anti-ERBB2 (Vector Laboratories, Inc, CA). The dilution of each antibody was according to the manufactures’ instructions, and positive staining was detected using diaminobenzidene (DAB) (Vector Lab, CA) according to the manufacturer's instructions. The data was independently reviewed by two pathologists.

### Reverse transcription-PCR (RT-PCR) and quantitative real-time PCR (Q-PCR)

The total RNA from tumor tissues or organs was isolated using the RNeasy micro kit (#74004, QIAGEN) according to the manufacturer’s instructions. Subsequently, cDNA was synthesized by reverse transcription (RT) with ThermoScript™ RT-PCR system (Invitrogen) per the manufacturer’s instructions and followed by PCR. The primers used were as follows: AKT: 5’TCCTCAAGAAGGAAGTCATCGT-3’ (forward) and 5’-CGTACTCCATGACAAAGCAGAG3’ (reverse); myr-Akt1: 5’- ACCACTTGTCTCACATCCTTGTT -3’ (forward) and 5’TTCTAGACTTGGGCTTGCTCTT-3’ (reverse); β-actin: 5’- GTCTTCCCCTCCATCGT-3’ (forward) and 5’- CGTACATGGCTGGGGTGT-3’ (reverse). The PCR products were separated on 2% agarose gels with ethidium bromide. The final results for each gene were quantified using GelQuant.NET software (BiocheLabSolution.com) and adjusted for β-actin. Q-PCR analysis was performed with iCycle iQ real-time PCR detection system (Bio-Rad Lab, Hercules, CA) using SYBR Green Master Mix (#204143, QIAGEN). The primers used were as follows: SLUG: 5- 5’-AGAGCATTTGCAGACAGGTCA-3’ (forward) and 5’AGCAGCCAGATTCCTCATGTT-3’ (reverse), 18S, 5'-GATCCATTGGAGGGCAAGTC-3' (forward) and 5'-TCCCAAGATCCAACTACGAG-3' (reverse). The mRNA levels of SLUG were quantified by measuring the threshold cycle (Ct) and were adjusted for the level of 18S.

### Mammary gland whole mounts

Mammary glands near the hind legs were harvested from WT and transgenic mice at the indicated times and fixed in 10% formalin overnight. The fixed mammary glands were then placed in 75% ethanol for 2 hours and placed in acetone overnight at -20°C. The tissues were then rehydrated with successive incubation with different concentrations of ethanol, stained with hematoxylin for 1.5 hours, and then rinsed in crude tap water overnight. Tissues were then placed in 50% ethanol with 12 N of HCl for 30 minutes for destaining followed again with successive incubation in graded ethanol for dehydration. Subsequently, the tissues were incubated in xylene, then mounted in Permount (Fisher Scientific). Under 10x magnification, the total number of buds (terminal end buds and alveoli buds) were counted and divided by the total number of ducts as follows: pre-puberty and pubertal mice 2-4 ducts, 12-week virgin mice 7-11 ducts, 16-week and 26-week mice 11-17 ducts. Two mice per condition and per genotype were used for analysis.

### Western blot analysis

The total protein from snap-frozen tumor tissues were extracted by homogenization using the Powergen Homogenizer 125 (Fisher Scientific) in 1 ml extraction buffer (25 mM Tris-HCl pH 7.6, 150 mM NaCl, 1% NP-40, 1% sodium deoxycholate, 0.1% SDS and 10 μl Protease Inhibitor Cocktail - Cat#78410, Thermo Scientific). Homogenates were centrifuged at 1000 g for 10 minutes at 4°C, and 80 μg of proteins for each sample were used for Western Blot analysis. The following antibodies were used: anti-phospho-Akt1 (ser473), anti-AKT, anti-Cyclin D1 (Cell Signaling, MA); anti-ERα, anti-CK18, anti-Twist, and anti-β-actin (Santa Cruz Biotechnology, CA).

### Measurement of estradiol levels

Blood was collected from both WT and transgenic mice from each of the following conditions: 3 month-old virgin mice, ~4 month-old lactating mice 3 days after giving birth, and ~ 5 month-old post-lactating mice one month after giving birth. The blood samples were collected immediately after euthanization (two mice for each group). Serum estradiol (E2) levels were measured by ELISA assay (Cat# ES180S-100, Calbiotech Inc, CA) per the manufactures’ instructions. The E2 level was determined based on the principle of competitive binding between E2 in serum samples and E2 enzyme conjugate for a constant amount of anti-estradiol antibody. The sensitivity of the assay is <3 pg/ml.

### Statistical analysis

Statistical analysis was performed with the SPSS statistical package (Version 11.0 for windows, IBM). Kaplan-Meier survival curve analysis with the log-rank test was used to determine the tumor-free survival between transgenic and wild-type mice treated with DMBA. The Spearman rank test was used to examine the differential incidences of different tumors types between different groups of DMBA treated mice. P-values < 0.05 were considered statistically significant.

## Results

### MMTVmyr-Akt1 transgene expression in transgenic mice

To determine the organ specificity of MMTV driven myr-Akt1 transgene expression, we extracted RNA from different organs of the female mice at different ages. As shown in Figure 1A, myr-Akt1 was detected in the mammary glands, the uterus, the ovaries, and the heart of virgin transgenic mice at 9 weeks old as well as post-lactating transgenic mice at 16 weeks old. The data in Figure 1B showed mRNA levels of myr-Akt1 expression at different development stages of transgenic mice. The mRNA level was detected in the mammary gland, but not in the other organs of 4 week old virgin mice. The expression of MMTVmyr-Akt1 in the mammary glands of transgenic mice significantly increased in the lactating stage 3 days after giving birth and decreased at the post-lactation stage one month after giving birth. The myr-Akt1 expression in the lungs, the heart, the uterus and the ovaries began to be detected at 9 weeks in the virgin transgenic mice. The myr-Akt1 in the uterus and ovaries were also significantly increased during pregnancy and lactation (Figure 1B). In contrast, myr-Akt1 was undetectable in WT mice in the same organs, at varying ages, and lactation stages (data not shown). The myr-Akt1 dominant phenotype in the virgin transgenic mice was exhibited until 12 weeks. A clear increase in the phosphorylation of Akt1 at ser473 (pAkt1) was detected by IHC analysis in the mammary glands of 12-week-old virgin female transgenic mice, but not in the young 4-week-old virgin transgenic mice (Figure 1C). Neither the 12 week-old nor the 4-week-old WT mice had pAkt expression in their mammary glands. In addition, the serum estradiol (E2) levels in the transgenic mice were significantly higher during the lactating stage and remained higher even in the post-lactation stage compared to WT mice (Figure 2A). The levels of Akt1 expression followed a similar trend as E2 expression during the lactating stage (Figure 2B). Interestingly, the total AKT levels in the mammary glands of the virgin transgenic mice at 5 weeks old, at 9 weeks old, and during lactation were significantly higher compared to WT mice at the same mammary development stages. The total AKT levels in the liver, the lungs, the ovaries, and the uterus of the WT and MMTVmyr-Akt1+ mice also increased significantly during the multiparous/lactation period and decreased at the post-lactation stage a month later after birth (Figure 2C). Overall, transgenic mice had higher total AKT expression in their organs compared to WT mice (Figure 2C and Additional file 2: Figure S2).

**Figure 1:** **Expression of activated Akt1 in transgenic mice at different development stages. (A)** Total RNA was extracted from the indicated organs of virgin (9 week old) and post-lactating (16 week old) transgenic mice. RT-PCR was performed with primers for myr-Akt1 and β-actin. Three mice per genotype, per age group were used for analysis. Myr-Akt1 was detected in the lungs, heart, uterus, and mammary glands of the virgin and post-lactating mice. **(B)** The mRNA levels of myr-Akt1 were quantified in different organs of the transgenic mice at different developmental states. Myr-Akt1 levels were adjusted for the levels of β-actin. Data are presented as bar graphs. The bars indicate mean levels and SD from three mice and “*” indicates p < 0.05 compared to the virgin mice. **(C)** H&E staining (a and b), and immunohistochemical detection of phospho-Akt1 (ser743) (c and d) in the mammary glands of wild-type mice (WT) and transgenic mice (MMTVmyr-Akt1).

**Figure 2:** **Estradiol level and total AKT expression in wild-type (WT) and transgenic mice. (A)** Blood samples were collected from virgin, lactating, and post-lactating mice and serum estradiol levels were measured by ELISA assay according to the manufacturer’s instructions. The line graph indicates trend of estradiol levels (mean of seven samples plus SD) in WT (n = 21) and transgenic mice (n = 21) from virgin to post-lactating stage. **(B)** RNA was collected from the mammary glands of WT and transgenic mice and RT-PCR was performed with AKT primers and quantified with β-actin. The lines indicate the trends of mean levels of total AKT adjusted for β-actin in the mammary glands of WT (n = 9) and transgenic mice (n = 9) at pre-puberty virgin (5 weeks olde, n = 3), puberty virgin (9 weeks olde, n = 3), lactating (14 weeks old, n = 3) and post-lactating (16 weeks old, n = 3) stages. **(C)** mRNA levels of total AKT from different organs in WT (top) and transgenic mice (bottom) at indicated stages were determined by RT-PCR. The mean total AKT levels are adjusted for β-actin was shown in the bar graphs. Each bar indicates mean and SD from four mice. Each sample was triplicated and “*” indicates p < 0.05 compared to virgin.

To understand the effect of Akt1 activation in mammary gland growth, whole mounts of mammary glands from different ages and stages of transgenic mice were compared to WT mice at the same ages and stages. The assessment compared mice at the pre-pubertal stage (10 day old pups), pubertal stage (3 week old virgins), post-pubertal stage (12 week old virgins), and among the post-lactation stage (16 week old, 2 weeks after weaning and 26 week old, 12 weeks after weaning). The mammary structure and cellular composition were similar between younger virgin MMTVmyr-Akt1+ mice and WT mice. Differences included fewer ducts with end buds (characterized as conspicuous club-shaped structures) [18] growing from fewer terminal branches (Figure 3Aa, 3Ab and 3Af, 3Ag). A significant difference was observed in 12 week old virgin mice group. The mammary glands from the MMTVmyr-Akt1+ mice showed a marked increase in the number of terminal branches and terminal end buds (TEB) compared to WT mice (Figure 3Ac and 3Ah). It is well known that the alveolar epithelium expands during pregnancy and undergoes apoptosis and remodeling during involution [19]. However, the alveoli buds which are smaller and hollow cavities, were observed in the mammary glands of the MMTVmyr-Akt1+ mice 2 weeks after weaning, but not in the WT mice (Figure 3Ad and 3Ai). Even after 3 months of weaning, there were still fewer alveoli structures in the MMTVmyr-Akt1+ mice (Figure 3Ae-3Aj and 3B). These data indicate a delayed involution due to the activation of Akt. In addition, the number of terminal end buds and alveoli buds in the mammary glands were quantified throughout development. Figure 3C demonstrates that the number of total buds were slightly more in the MMTVmyr-Akt1+ mice than in the WT mice. There were no statistically significant differences among the 10 day old and 3 week old mice. However, activation of Akt played a crucial role in the development of buds during the post-pubertal period. The total numbers of buds were significantly more in the MMTVmyr-Akt1+ mice at 12 weeks old compared to the WT mice (Figure 3C).

**Figure 3:** **Effect of myr-Akt1 in mammary gland development**. Representative whole mounts of WT **(Aa to Ae)** and myr-Akt1+ **(Af to Aj)** mammary glands at the indicated ages and stages. Black arrows indicate ducts. Blue arrows indicate side branches and green arrows indicate terminal end bubs (TEB). **(B)** An enlarged example of duct and alveolar buds from mammary glands of 26 week old myr-Akt1+ mice (12 weeks after weaning). **(C)** Quantification of the average number of buds per duct in the indicated ages and stages of WT and myr-Akt1+ mice. The numbers of bubs were counted and divided by the total number of ducts in the fields. Five fields per mouse were counted in the 12 week, 16 week and 26 week age groups. Two mice per age group and per genotype were used for analysis. The data represented in line plot is mean ± SD and “*” indicates p < 0.05 compared to WT mice at same age.

### Reproduction and survival rate of mice carrying myr-Akt1 transgene

The survival rate of litters was similar between transgenic and WT mice (Table 1). Comparing to litters from MMTVmyr-Akt1+/- parents, the survival rate was slightly higher in litters from MMTVmyrAkt1+/+parents (96% vs. 88%). The average babies per litter were also similar among the transgenic and the WT mice (Table 1). In addition, the body weight was slightly higher in the transgenic mice compared to the WT mice (Additional file 3: Figure S3).

**Table 1:** Survival rates of information of transgenic mice

**Generation**	**MMTV-myr-Akt1**^**+/+**^			**MMTV-myr-Akt1**^**+/-**^			**MMTV-myr-Akt1**^**-/-**^	
	**Survival Rate of litters (%)**	**Average pups per litter (range)**	**Myr-Akt + pups (%)**	**Survival Rate of litters (%)**	**Average pups per litter (range)**	**Myr-Akt + pups (%)**	**Survival Rate of litters (%)**	**Average pups per litter (range)**
**F1**	-	-	-	88	7 (4-8)	57	78	9
**F2**	100	8 (7-9)	61	96	7 (6-7)	35	-	-
**F3**	100	5 (3-7)	53	90	6 (3-9)	43	100	7
**F4**	97	6 (3-8)	57	88	8	14	95	6 (5-8)
**F5**	100	7 (4-9)	31	68	7 (2-8)	53	-	-
**F6**	95	7 (6-10)	29	96	8 (6-9)	37	100	8 (6-9)
**F7**	94	6 (2-9)	37	94	7 (2-9)	27	95	7 (4-8)
**F8**	88	8 (7-9)	36	82	7 (3-10)	22	100	7 (6-7)
**Average**	96	7 (2-10)		88	7 (2-10)		95	7 (5-9)

### Development and pathology of tumors induced by DMBA in MMTVmyr-Akt1 mice

Previous studies have shown that AKT1 transgenic mice expressing constitutively active Akt1 have delayed mammary gland involution, but do not exhibit neoplasia [13,14]. Formation of mammary neoplasms requires induction by a carcinogen. In this study, 28 mice (14 MMTVmyr-Akt1+ and 14 WT) were followed until 18 months of age. No spontaneous malignant neoplasms were observed in the mammary glands or the other organs of mice with and without the MMTVmyr-Akt1 transgene (data not shown). The transgenic and WT female mice at the virgin stage and at post-lactation a month after giving birth were fed by oral gavage with 1 mg doses of DMBA once a week for 6 consecutive weeks. The ages of virgin mice were between 14 to16 weeks old, and between 20 to 22 weeks old among the post-lactation mice. The sequence of DMBA treatments is shown in Figure 4A. The earliest tumors were detected 12 weeks after the completion of DMBA treatment. Figure 4B shows an example of tumor growth in the mammary glands of transgenic mice. The oral DMBA treatment induced mammary tumors and tumors in other organs as well. There were no significant differences in the death rate between the WT and the MMTVmyr-Akt1+ mice (Figure 4C). Overall, the incidence of mammary gland malignant tumors and benign masses were significantly higher in the MMTVmyr-Akt1+ mice in the WT mice (42.9% vs. 7.1%) as shown in Figure 4D (left).

**Figure 4:** **Tumor development in wild-type and MMTVmyr-Akt1 transgenic mice treated with DMBA. (A)** Experimental design and scheme of DMBA treatment. **(B)** Mammary gland tumor growth in transgenic mouse. **(C)** Tumor-free survival curves in wild-type and MMTVmyr-Akt1 transgenic mice, analyzed by Kaplan-Meier survival curve analysis with log-rank test. **(D)** Bar graphs indicate incidences of tumor formation in wild-type (WT) and transgenic mice (MMTVmyr-Akt1) (left), and incidences of mammary gland tumors and other site tumors in transgenic mice from MMTVmyr-Akt1 ^+/+a^nd MMTVmyr-Akt1 ^+/-^groups (right). At left, p = 0.009 indicates the significant differences in the incidence of mammary tumor and other organ site tumor formation among WT and myr-Akt1 mice. At right, “*” indicates p < 0.05 between the indicated two groups and "^" indicates p < 0.01 between the indicated two groups.

Detailed histopathological descriptions of the DMBA induced tumors in WT and transgenic mice are shown in Table 2. Overall 32.1% of the MMTVmyr-Akt1+ mice developed mammary carcinomas. Approximately 22% of the myr-Akt1 driven mammary tumors induced by DMBA were infiltrating poorly differentiated carcinomas and had malignant bone lesions in the same mice. The malignant bone lesions showed similar pathology as the mammary carcinomas from the same mouse. The incidence of mammary carcinomas in the MMTVmyr-Akt1+/+mice were significantly higher than in the MMTVmyr-Akt1+/- mice (35.3% vs. 27%, p < 0.05) (Figure 4D, right). The incidence of benign mammary masses were higher in the MMTVmyr-Akt1 +/- mice compared to MMTVmyr-Akt1+/+mice. In addition, the MMTVmyr-Akt1 +/- mice induced with DMBA also developed tumors at other sites. Interestingly, DMBA induced mammary gland tumor formation in virgin and post-lactating transgenic mice, but not in post-lactating WT mice (Table 3). Table 3 demonstrates that approximately 23.5% and 45.5% of mammary gland malignant lesions were induced by DMBA in virgin and post-lactating transgenic mice, respectively. DMBA also induced salivary gland and lung carcinomas in WT virgin mice. The benign mammary lesions also appeared in MMTVmyr-Akt1+ mice treated with DMBA at virgin and post-lactation stages, but did not appear in the WT mice. In addition, DMBA treatment induced carcinomas in the stomach and benign skin lesions in both the WT and transgenic mice. The incidence of mammary gland tumor formation in post-lactating transgenic mice was concordant with relatively higher expression levels of pAkt and total AKT in the mammary gland tissues as shown in Figures 1 and 2. The expression of myr-Akt1 in the ovaries of the transgenic mice may result in increased circulating estrogen levels. There may be a feedback loop between AKT pathway and estrogen pathway which is enhanced during carcinogen-induced tumorigenesis.

**Table 2:** Incidence and histopathological description of malignant and benign tumors induced by DMBA

	^WT (N = 28) N (%)*	^^Myr-Akt1 + (N = 28) N (%)*
Infiltrating poorly differentiated mammary carcinoma with bone metastases	0	2 (7.1%)
Poorly differentiated mammary carcinoma with necrosis	2 (7.1%)	7 (25.0%)
Salivary gland carcinoma with bone metastasis	1 (3.6%)	0
Carcinoma in the wall of the stomach	1 (3.6%)	1 (3.6%)
Carcinoid pattern of malignancy in lung	1 (3.6%)	0
Benign lesions of mammary gland with lymploid tissue	0	3 (10.7%)
Endometrial cystic changes with focal hyperplasia	1 (3.6%)	0
Benign squamous epithelium tumor	1 (3.6%)	1 (3.6%)

^Wild-type mice.

^^MMTV-myr-Akt1 transgenic mice.

*The percentages correspond to the total number of treated mice.

**Table 3:** Incidence of malignant and benign tumors induced by DMBA

	**Wild-Type (N = 28)**		**MMTV-myr-Akt1 + (N = 28)**	
	**Virgin (N = 17)**	**Post-lactating (N = 11)**	**Virgin (N = 17)**	**Post-lactating (N = 11)**
Mammary carcinoma	2 (11.8%)	0	4 (23.5%)	5 (45.5%)
Salivary gland carcinoma	1 (5.9%)	0	0	0
Stomach carcinoma	1 (5.9%)	0	0	1 (9.1%)
Malignancy in lung	1 (5.9%)	0	0	0
Benign mammary tumor	0	0	2 (11.8%)	1 (9.1)
Endometrial hyperplasia	1 (5.9%)	0	0	0
Benign skin tumor	1 (5.9%)	0	0	1 (9.1)

### Phenotype of mammary malignant tumors

The phenotype of the mammary tumor tissues from WT and transgenic mice were further characterized and distinctive differences were identified. The mammary tumors from positive transgenic mice were more likely to have activation of Akt1 and to be ER + and/or PR+, HER2- and EGFR+. DMBA-induced mammary gland tumors from WT mice were negative for pAkt expression and expressed lower levels of ER and PR. EGFR expression was moderately positive whereas HER2 expression was negative. Positive Ki67 expression was identified in all the mammary tumors from transgenic mice. Among the WT mice, ~60% of tumors were positive for Ki67 (data not shown). The tumors that had higher Ki67 expression were more likely to be PR+. HER2 receptor expression was not detected in any of the tumors (data not shown). The IHC data in Figure 5A shows examples of protein expression for pAkt1, ERα, and EGFR in tumors from the transgenic (P1) and WT (N2) mice. The association between pAkt1 overexpression and increased nuclear expression of ERα in mammary gland tumor from mouse-P1 is demonstrated in Figure 5A. The malignant bone lesions from transgenic mice, P1 and P3, were also correlated with ERα positive tumors (data not shown). Moderate to high expression of EGFR was observed in DMBA-induced mammary tumors from both transgenic and WT mice. Interestingly, the EGFR expression was mainly in the cytoplasm of the tumor tissues from transgenic mice and in the cell membrane of the tumors from the WT mice (Figures 5A, d and h). The expression of pAkt in relation to ERα expression in transgenic mice was also confirmed by western blot analysis (Figure 5B). Malignant mammary tumors from transgenic mice (P1, P2, and P3) had increased pAkt1 and strong ERα expression while tumors from WT mice (N7 and N2) had lower or undetectable pAkt1 and weak expression of ERα. The total AKT levels remained similar in all tumors from transgenic and WT mice (Figure 5B).

**Figure 5:** **Characterization of malignant mammary tumors. (A)** H&E staining (a and e) and immunohistochemical analysis were used to determine the level of phospho-Akt1 (pAkt ser473) (b and f), ERα (c and g), and EGFR (d and h) expression in mammary tumors from wild-type mouse (N2) and MMTVmyr-Akt1 transgenic mouse (P1). The arrows indicate positive staining. **(B)** Protein was extracted from the mammary tumors and western blot analysis was used to determine the indicate protein expression. **(C)** RNA was extracted from mammary carcinomas from four transgenic mice and two wild-type mice. RT-Q-PCR was performed with the indicated primers. The bar graph indicates relative expression levels of the indicated genes adjusted for 18S from the four transgenic and two wild-type mice. Each bar indicates mean and SD of three individual tests. “*” indicates p < 0.05 between the two groups for the indicated genes. **(D)** RNA samples from mammary tumors of transgenic mice (P1, P3, and P7) and wild-type mice (N7 and N2). RT-Q-PCR was performed to quantify levels of slug. The bars indicate relative levels of slug adjusted for 18S expressed in the mammary malignant tumor samples from the indicated mouse. Each bar indicates mean and SD of three individuals test. “*” indicates p < 0.05 compared to N2 and N7 respectively.

### Cyclin D1 and EMT marker twist and slug expression in mammary tumors from MMTVmyr-Akt1 mice

It is well known that active Akt1 induces cell proliferation. Cyclin D1 is one of the key cell cycle regulators and has been implicated in oncogenesis. In our model, Cyclin D1 expression levels varied in mammary tumors from transgenic mice but were overall lower in tumors from WT mice (Figure 5C). However, the Cyclin D1 expression level determined by western blot analysis did not fully correlate with Ki67 expression as determined by IHC analysis (data not shown). Data in Figure 5C shows increased AKT and decreased PTEN mRNA levels in tumors from mice carrying the myr-Akt1 transgene.

Furthermore, the EMT markers, twist and slug, were up-regulated by the myr-Akt1 transgene. Previous studies have shown that increased invasiveness and motility are correlated with the mesenchymal phenotype [20]. In our model, mice which carried the myr-Akt1 had higher slug and twist expression in the mammary tumors and were more likely to have tumors with invasive and metastatic characteristics. Evaluation of tumor pathology revealed that the mammary tumors from the transgenic mice, P1 and P3, were poorly differentiated infiltrating carcinomas with bone metastases. Concordantly, twist (Figure 5B) and slug (Figure 5D) were highly expressed in the tumors from P1 and P3. The WT mouse, N7, had a poorly differentiated mammary carcinoma and carcinoid pattern of malignancy in the lung. These malignant lesions also had increased twist expression as well as relatively higher expression level of slug (Figure 5C and 5D). Pan-CKs and CK18 expression was also evaluated in these mammary tumors. The epithelial marker, CK18, protein level expression was significantly high in all mammary tumors from transgenic and WT mice (Figure 5B). The benign mammary masses also expressed CK18 protein but the levels were lower compared to the malignant mammary tumors (data not shown). The overall pan-CK expression was also higher in malignant mammary tumors from transgenic mice than tumors from WT mice (data not shown).

## Discussion

The goal of this study was to examine the oncogenic role of Akt in the development of mammary tumors. Myristoylation of Akt is a well-accepted mechanism to produce constitutively activated Akt in cells. Hence, we selected an established DNA structure of constitutively active Akt1 (myr-Akt1) that was generated by Upstate Biotechnology and tested *in vitro* in our previous study [12]. Myr-Akt1 was driven by MMTV-LTR to target the expression of the transgene specifically to the mammary gland tissue. Similar strategies have been used by other groups to develop Akt1-transgenic mouse models [13,15].

The myr-Akt1 transgene was expressed most significantly in the mice mammary glands in our model. This is consistent with the findings that there is an increase in the MMTV-LTR transcriptional activity throughout mammary development and during pregnancy [21]. Increased phosphorylation of Akt at ser473 was detected in the mammary glands of 9 week old transgenic mice in the model developed by Blanco-Aparicio and colleagues [15]. Similarly, we detected phosphorylated Akt at ser473 in our transgenic mice at 12 weeks old. Myr-Akt1 was also detected in the brain, salivary glands, ovaries, and uterus in the model developed by Blano-Aparicio group. We also found expression of myr-Akt1 in the ovaries and uterus of our transgenic mice. We did not examine expression in the brain or salivary glands in our study. In addition, the mRNA level of total AKT was higher in most organs from our transgenic mice compared to wild-type mice examined at pre-puberty, puberty, during lactation, and at post-lactation stages.

In our model, a significantly high level of circulating estradiol remained in the transgenic mice at during the later stages of lactation and decreased at the post-lactation stage. Overall transgenic mice had higher estradiol levels compared to WT mice. Estradiol is mainly produced by the granulosa cells of the ovaries. Under normal physiological conditions during pregnancy, circulating estrogen increases and decreases during the lactation period. However, activation of Akt1 in the ovaries may increase the proliferation of granulosa cells and lead to an increased production of estradiol even in the later-lactation stage. The higher circulating estrogen levels could further induce higher AKT expression. The increased estradiol by the activation of Akt1 in the ovaries could partially contribute to the mammary tumorigenesis in the transgenic mice in our model. Further studies examining mice with removed ovaries need to be conducted for clarification. However, the mammary tumorigenesis is more likely to be driven by the expression of myr-Akt1 in the mammary glands since we did not observe any ovarian or uterine cancers in our model. In addition, local estrogen biosynthesis such through Akt1 mediated aromatase expression in the mammary glands or myr-Akt1 induction of prolactin [22-24] could all contribute to mammary tumorigenesis. High levels of prolactin have been associated with postmenopausal breast cancer risk [25].

In our model, the transgene was maintained in C57BL6 mice which are genetically resistant to spontaneous mammary tumor formation [15,26] in order to reduce background tumor activity in the wild-type mice. Therefore, there is no spontaneous tumor formation in the wild-type mice in this study.

The role of Akt1 in mammary gland development and function has been examined in the postnatal stage of mice. The activation of Akt1 or overexpression of total AKT has been shown to delay mammary gland involution, and to induce hyperplasia in similar Akt1-transgenic mouse models [13,14]. In this study, we further examined the role of Akt1 in mammary gland development from pre-puberty, puberty, post-puberty (virgin), lactating to post-lactation stages. Our data showed for the first time that myr-Akt1 played a crucial role in the development of the early adult mammary gland. Myr-Akt1+ mice had mammary ductal outgrowths though the fat pads and extending alveolar epithelium during the post-puberty stage. Consistent with other Akt1 transgenic models, a delayed mammary gland involution was observed in our model as well. The activation of Akt has been shown to accelerate mammary tumorigenesis in MMTV-c-ErbB2 mice [27]. However, overexpression or activation of Akt1 in the mammary glands alone is not enough to induce dysplasia or neoplasia [28-31]. Activation of Akt1 induces oncogenic transformation upon exposure to carcinogens [15]. Similarly in our model, we demonstrated that exposure to the carcinogen DMBA in transgenic mice with active Akt1 expression led to a significantly higher incidence of mammary carcinoma. In addition we compared tumor formation between transgenic mice and WT mice at different ages.

Epidemiological studies have suggested that lactation may have some protective effect on breast cancer risk in humans [29-31]. Pregnancy and breast feeding have been associated with a reduction of lifetime risk of breast cancer among premenopausal women and women with family history of breast cancer [32-34]. Mechanism studies using mouse models suggest that the secretory mammae and low rate of DNA synthesis in lactating mammary glands may account for the elimination of carcinogens [35-37]. Studies have found that lactating mice were relatively refractory to the effects of chemical carcinogens. Conversely, the levels of estrogen and prolactin are increased during pregnancy and lactation, and the high levels of estrogen and prolactin could be associated with the development of breast cancer [25,35]. Normally, the mammary gland regresses to its pre-pregnancy status by a coordinated process of apoptosis, remodeling, and inflammation following pregnancy and lactation [38]. Activation of Akt in mammary tissue could result in de-regulation of the survival signal [31]. The normal mammary gland involution after pregnancy and lactation could be interrupted by active Akt1 expression in mammary tissue. The irregular involution of the mammary gland might increase susceptibility to carcinogen-induced tumor formation. Data from our current study demonstrated that the mice carrying the myr-Akt1 transgene in the mammary glands had accelerated carcinogen-induced tumorigenesis during the virgin and post-lactation stages. The protection against carcinogen-induced mammary malignancy by lactation was eliminated by expressing active Akt1 in the mammary tissues of the transgenic mice. We found that there was no DMBA induced tumor formation in the wild-type mice throughout pregnancy and lactation. However, DMBA induced mammary carcinomas were observed in 45.5% of mice with the MMTVmyr-Akt1 transgene.

Our studied identified that the DMBA induced mammary carcinomas in both transgenic and wild-type mice were poorly differentiated. However, the tumor tissues from transgenic mice had increased phosphorylated Akt1 at ser473 and the tumors showed strong positive expression of nuclear ERα. These findings are similar to data reported from another group [15]. The tumors from our model were also positive for EGFR expression. Moreover, the tumors with low ERα expression concurrently had membranous expression of EGFR. ERα positive tumors with increased pAkt were associated with strong cytoplasmic expression levels of EGFR. However, the function of cytoplasmic expression of EGFR is unclear, although both membranous and cytoplasmic expression of EGFR has been reported before in cancers such as pancreatic cancer. Tissues resected from pancreatic cancer patients with EGFR over-expression in the cell membrane showed worse clinical outcomes compared to patient tissues with low EGFR expression [39]. Other studies demonstrated that EGFR expression in the membrane is more strongly associated with malignant tumors, while cytoplasmic EGFR expression is associated with normal cells or benign tumors [40,41]. Cytoplasmic EGFR over-expression was not significantly associated with recurrence or survival in our study.

It has been suggested that the activation of Akt might cooperate with ERα activity in the development of mammary tumors induced by DMBA [15]. The observations from our current study are in agreement with this Akt - ERα cooperation concept. In addition, our data implies that the Akt-ERα cooperation may also have interactions with the EGFR pathway. Cyclin D1 plays role in tumor cell proliferation and is inversely correlated with tumor size in human breast cancer [42]. Overexpression of Cyclin D1 has been reported in 40% to 90% of invasive breast cancers, while gene amplification is seen in about 5–20% of tumors [43]. Increase in the protein levels of Cyclin D1 is apparent in hyperplasias and is further increased in malignancies [43,44]. Cyclin D1 has also been shown as an essential oncogenic intermediary for the *Neu* pathway by inducing mammary carcinoma in transgenic mice [28,45]. In our model, we observed that Cyclin D1 expression was higher in DMBA-induced myr-Akt1 driven mammary carcinomas. However, Cyclin D1 expression was not simply associated with activation of Akt1. It was also not essential for ER-positive tumor formation since the levels of Cyclin D1 varied in tumors from the transgenic mice. Similar observations were reported by Blanco-Aparicio et al. [15].

In humans, more than 60% of breast cancer is ERα-positive. Endocrine therapy, tamoxifen, is the most important systemic treatment of ER-positive breast cancer. Unfortunately, patients with advanced ER-positive disease eventually acquire resistance to tamoxifen treatment. The MMTVmyr-Akt1 transgenic mice tumor formation induced by carcinogens could mimic ER-positive human breast cancer, as shown with increases in pAkt, Cyclin D1, and EGFR. Furthermore, the transgenic mice in our model exhibited characteristics of advanced ER-positive mammary tumors with bone metastasis and increased expression of the mesenchymal markers, twist and slug. The data from this study showed that mammary tumors with metastatic characteristics were associated with increasing expression of twist and slug. The bone metastatic lesions were also positive for ERα. Therefore, the MMTV-myr-Akt1 transgenic mice could be useful for exploring the underlying mechanisms of ER-positive breast cancer acquiring resistance to tamoxifen and developing metastatic disease. EGFR*-*targeted therapy, such as cetuximab and lapatinib in combination with hormonal therapy may also be explored as methods to overcome resistance. Patients with ERα-negative or triple negative breast tumors frequently demonstrate increased EGFR expression [46,47]. These patients are more likely to have poor disease outcomes. Similar to the aforementioned patient-based studies, we observed that wild-type mice with mammary tumors from DMBA induction showed an inverse relationship between nuclear expression of ERα and membranous EGFR. Thus, the carcinogen-induced mammary tumors from virgin mice in this study might also provide an *in vivo* model for better understanding the etiology and tumor biology of this type of breast cancer. From a translational perspective, this will facilitate the design of better target therapies for treating ER/HER2-/EGFR + breast cancer.

## Conclusions

In summary, data from this study suggest that activation of Akt1 in mammary tissue increases the risk of developing mammary tumors through carcinogen induction. The breast cancer risk reduction associated with breast feeding could be attenuated by the activation of Akt1 in the mammary tissues. These data further affirm that our MMTVmyr-Akt1 transgenic mouse is a valuable resource for understanding the mechanisms of ER + breast cancer development.

## Abbreviations

myr-Akt1: myristoylated-Akt1; DMBA: 7, 12 dimethyl-1,2-benzanthracene; MMTV-LTR: Mouse Mammary Tumor Virus Long Terminal Repeat Promoter; CMV: Cytomegalovirus immediate-early promoter; E2: Estradiol; EGFR: Epidermal growth factor receptor; ER: Estrogen receptor; PR: Progesterone receptor; HER2: Human Epidermal Growth Factor Receptor 2; EMT: Epithelial-mesenchymal transition.

## Competing interests

The authors declare that they have no financial and non-financial competing interests.

## Authors’ contributions

JVV made contributions to conception, design, overall guidance for the study, data interpretation and manuscript editing, revising for important content; YW made contributions to design the transgene and experiments; data acquisition, analysis, interpretation, and drafting the manuscript; JK made contributions to acquisition, analysis of the data and also involve the manuscript preparation, MS made contributions to the preparation of the manuscript; and YE made contributions to analysis and interpretation of the data, as well as preparation of the manuscript. All authors read and approved the final version of the manuscript to be published.

## Pre-publication history

The pre-publication history for this paper can be accessed here:

http://www.biomedcentral.com/1471-2407/14/266/prepub

## Supplementary Material

Additional file 1: Figure S1 The myr-Akt1 transgene and integration of the transgene in transgenic mice. The CMV promoter in myr-Akt1 DNA structure (#21-151, Upstate Biotechnology) was replaced by MMTV-LTR **(A)** and the construct was digested and the fragment containing MMTV-LTR promoter. Myr-Akt1 sequences and SV40 polyadenylation signal were isolated and purified **(B)**. **(C)** Shows the copy number standard curve of qPCR. The simple linear regression standard curve was built with logarithm transformed serial diluted myr-Akt1 plasmid DNA (from 0.01 copies to 100 copies as described in methods) as an independent variable, and qPCR Ct numbers as a dependent variable. **(D)** DNA from transgenic mice and WT mice was amplified by q-PCR and the numbers of transgene copies were estimated by the copy number standard curve according to the numbers of Ct for each sample. Each sample was triplicated and the bar indicates mean ± SD. Click here for file

Additional file 2: Figure S2 Expression of Akt1 in wild-type (WT) and transgenic mice (MMTV-myr-Akt1). Total RNA was extracted from indicated organs of virgin (A) (9 weeks) and post-lactating (B) (16 weeks) WT and transgenic mice. Three mice per genotype, per age group were used for analysis. RT-PCR was performed with primers of Akt1 and β-actin. Click here for file

Additional file 3: Figure S3 Growth of wild-type and transgenic mice. Body weight of wild-type (WT) mice and transgenic mice (MMTV-myr-Akt1) were measured from F3 generation. The body weight was monitored from 1 month old of MMTV-myr-Akt1^+/+^, MMTV-myr-Akt1^+/-^ and WT mice until 6 months old. The body weight was mean of 6 to 8 per group and the SD was less than 2 percent of mean. Click here for file
